This article has been retracted.

# 8-bromo-7-methoxychrysin targets NF-κB and FoxM1 to inhibit lung cancer stem cells induced by pro-inflammatory factors

**DOI:** 10.7150/jca.30143

**Published:** 2019-08-28

**Authors:** Qing Yuan, Min Wen, Chang Xu, A Chen, Ye-Bei Qiu, Jian-Guo Cao, Jian-Song Zhang, Zhen-Wei Song

**Affiliations:** 1 Department of preclinical medicine, Medical College, Hunan Normal University, Changsha, 410013, China; 2 Department of Pharmaceutical Science, Medical College, Hunan Normal University, Changsha, 410013, China; 3 Key Laboratory of Study and Discover of Small Targeted Molecules of Hunan Province, Changsha 410013, China

**Keywords:** lung cancer, cancer stem cell, tumorigenesis, inflammatory factor, NF-κB, FoxM1

## Abstract

We have previously reported that 8-bromo-7-methoxychrysin (BrMC), a novel synthetic derivative of chrysin, was demonstrated anti-tumor activities against several human cancers, including lung cancer. Interaction between inflammation and cancer stem cell are recently increasingly recognized in tumorigenesis and progression. The purpose of this study was to investigate whether BrMC inhibits lung cancer stemness of H460 cells induced by inflammatory factors (TGF-β combined with TNF-α) and its potential mechanism. Our results showed that BrMC inhibited lung cancer stemness, as validated by enhanced self-renewal ability, higher* in vitro* tumorigenicity, and increased expression of CD133, CD44, Bmi1 and Oct4 in H460 cells administered TNF-α after prolonged induction by TGF-β, in a concentration-dependent manner. Both NF-κB inhibition by SN50 and FoxM1 suppression by thiostrepton (THI) prompted the inhibition of BrMC on lung CSCs. Conversely, overexpression of NF-κBp65 significantly antagonized the above effects of BrMC. Meanwhile, overexpression of FoxM1 also significantly compromised BrMC function on suppression of FoxM1 and NF-κBp65 as well as stemness of lung CSCs. Our results suggest that activation of NF-κB and FoxM1 by cytokines facilitate the acquisition CSCs phenotype, and compromise the chemical inhibition, which may represent an effective therapeutic target for treatment of human lung cancer. Moreover, BrMC may be a potential promising candidate for targeting NF-κB/ FoxM1 to prevent the tumorigenesis under inflammatory microenvironment.

## Introduction

Lung cancer is the leading cause of cancer-related death 1 and around 85% of new diagnosed lung cancer is non-small-cell lung carcinoma (NSCLC) 2. In spite of chemotherapy and targeted therapies available, a 5-year survival rate for NSCLC is only 18% 3-5. Therefore, further exploration of new therapeutic agents is necessary to improve therapeutic outcomes in NSCLC.

Many clinical evidences uncovered the etiological landscapes of lung carcinogenesis, among which the inflammation cytokines are contributing the risk to the development and subsequent progression 6, 7. Especially, exists data suggest that tumor necrosis factor-alpha (TNF-α) and transforming growth factor-beta (TGF-β) are both the most potent inducer of lung cancer promoting microenvironment 8, 9. Presence of TGF-β treatment potentiates the Epithelial-mesenchymal transition (EMT), which is a key step to early cancer metastasis 10. Remarkably, TNF-α can drive adaptive response to epidermal growth factor receptor (EGFR) inhibition in NSCLC, which is responsible for the resistance any failure of therapy in clinics 11.

Many studies have recently demonstrated that cancer stem cells (CSC) play a vital role in initiation and drive aggressive behavior in multiple cancers 12, 13, as while as lung CD133+ CSC constitute tumor-initiating activity in NSCLC 14, 15. Specially, this CSC characteristics, namely 'stemness', can be highly induced by chronic exposure to TNF-α combined with TGF-β 16, which is tightly involved by NF-κB signaling in cytokine production and immune responses. Recent discovery demonstrate NF-κB significantly involve the capability of CSCs 17 and is highly associated with poor survival in NSCLC 18. FoxM1 is a member of the forked box transcription factor family, which has been widely reported in regulating the stemness of CSC 19 and cause progression in tumorigenesis 20. Our previous data show that upregulation of FoxM1 expression promote the acquisition of CSC stem properties in NSCLC 21. Therefore, the NF-κB and FoxM1 are strongly associated with stemness of lung cancer, which may provide vital therapeutic targets in preventing human NSCLC.

Initiation and progression of tumorigenesis rely on the interaction of cancer stem cells with the tumor microenvironment 22, which are recruited by cytokine activity driven by inflammation or produced by cancer cells. Both TNFα and TGF-β have been shown to activate oncogenic pathway 23 and act on the NSCLC microenvironment 24. But, the acquisition of CSC features and consequent regulation on pathway derived from cytokine activity are still unclear. Our recent study demonstrated that 8-bromine-7-methoxychrysin (BrMC), a novel analogue of chrysin inhibits the malignant potential of cancer stem cells of hepatocellular carcinoma* in vitro* and *in vivo* 12. BrMC also can effectually reverse the M2 polarization of tumor associated macrophages by inhibiting NF-κB activation 25. For this reason, the purpose of this study was to evaluate whether BrMC can inhibit lung cancer stemness in H460 cells administered TNF-α after prolonged induction by TGF-β.

## Material and Methods

### Reagents

BrMC was synthesized according to previous described 26. The molecular formula is C_16_H_11_BrO_4_, the character is yellow like powder, the molecular weight is 347, and its purity is 99.5% by HPLC. BrMC was diluted with dimethyl sulfoxide (DMSO) to 10 mmol/L, the desired concentration was diluted to by DMEM medium before application. TGF-β and TNF-α from Sino Biological (Beijing,China). NF-κBP65 inhibitors (SN50) and FoxM1 specific inhibitors, thiostrepton (THI), are purchased from Sigma-Aldrich (St. Louis, MO, USA). NF-κBp65 antibody was purchased from Abcam (Burlingame, CA, USA). The Rabbit anti human β-actin monoclonal antibody was derived from Proteintech (Chicago, USA). The following antibodies were purchased from CST (Massachusetts, USA): Anti FoxM1, CD44, Oct4, CD133 antibodies. The recombinant adenovirus containing pHBad-MCMV-GFP plasmids and pHBad-MCMV-GFP-NF-κBp65 plasmids (virus titer: 10^10^pfu/mL, 2 mL) was prepared by Han Heng Biotech Corp (Shanghai, China). The FoxM1expressing lentivirus, ENi.s (enhanced infection reagents and Polybrene were purchased from Genechem (Shanghai, China), puromycin purchased from Jikai gene company, Catalog No.REVG0002, Shanghai, China. Opti-MEM reagent is the product of Invitrogen (China, Shanghai).

### Cell culture and Treatment

H460 cell line obtained from the Cell Bank of Chinese Academy of Sciences (China), were maintained according to previously described methods 27. For cell modeling, the cells were exposed to TGF-β (5 ng/mL) for 30 days followed by TGF-β (5 ng/mL) combined with TNF-α (5, 10 ng/mL) for 24 hours. For drug intervention, cells were administered BrMC at different amounts (1.0, 5.0 and 10.0 μmol/L) alone or BrMC (5.0μmol/L) plus SN50 (10.0 μmol/L) or BrMC (5.0 μmol/L) plus THI (10.0 μmol/L) for 24h. To explore mechanisms, H460 cells expressing NF-κBp65 or FoxM1 were treated with or without BrMC (5.0 μmol/L) for 24h.

### Cell transduction

For NF-κBp65 cDNA transduction, H460 cells grown in 24-well culture plates to 40-50% confluence were incubated overnight. Subsequently, they were infected with adenoviral particles packaged with control pHBAd-MCMV-GFP or pHBAd-MCMV-GFP-NF-κBp65 plasmids, respectively, cultured with Opti-MEM using the enhanced infection solution (ENi.s; GeneChem, China). Following 4h of transduction, DMEM containing 10% FBS was added to replace the transduction medium. The cells were then incubated for an additional 48h, prior to gene and protein level assessments. For stable expression of FoxM1 gene, H460 cells were infected with lentiviral particles containing full-length FoxM1 (NM_021953) or control vectors (GV358) using the enhanced infection solution (ENi.s; GeneChem, China). H460 cells stably expressing FoxM1 were isolated by puromycin selection.

### Sphere formation assay

Single-cells were seeded into ultra-low attachment 24-well plates (Corning, USA) at 10^3^ cells/ml in serum-free stem cell conditional medium. After a 6 day incubation period, spheroids were counted, to derive the sphere-formation rate by dividing the total number of spheres obtained by that of live cells seeded multiplied by one-hundred.

### Soft Agar Colony Assay

H460 cells administered TNF-α after prolonged induction by TGF-β were seeded into each 24-well plate in different conditions culture medium / agarose (at a 1:1 ratio) containing 1.2% agarose base layer and 0.7% agarose top layer. Cell culture the different conditions medium was removed and replaced periodically every 2 to 3 days. Following 12 days of incubation, cells were imaged under an inverted fluorescent microscope (Olympus, Japan). Individual stained colonies in each well were counted and the colony formation rate was calculated as follows: colony number / (number of cells seeded × each well efficiency), where each well is equivalent to the colony number divided by the number of cells seeded in the control medium.

### Western Immunoblot

Immunoblot was carried out according to a previous report 21.The primary antibodies used for membrane incubation targeted Bmi1, Oct4, CD133, CD44, NF-κBp65 and FoxM1. The membranes were further incubated with appropriate HRP-conjugated secondary antibodies. Immunoreactive bands were revealed by enhanced chemiluminescence. The UN-SCAN-IT software (Silk Scientific) was used for densitometry analysis, with β-actin serving as an internal reference.

### Statistical analysis

Experimental data were analyzed using SPSS 20.0 for Windows (SPSS Inc, Chicago, IL). Data representing mean ±SD were subjected to one-way ANOVA. First, the homogeneity of variance was determined. We used LSD to analyze pair wise comparisons among the groups. In the event of incomplete variance, the control and the experimental groups were analyzed with Tukey's test. A probability (P value) of less than 0.05 suggested statistical significance.

## Results

### Treatment of TGF-β combined with TNF-α promotes lung cancer stemness in H460 cells

To explore the association between cancer stem cell and inflammatory cytokines 28, a cell model was established by long term incubation of cytokines. NSCLC cell line H460 cells were exposed to TGF-β (5 ng/mL) for 30 days followed by TGF-β (5 ng/mL) combined with TNF-α (5, 10 ng/mL) for 24 hours. As shown in Supplementary Fig. 1, the incubated cells exhibited a typical morphological change of epithelial to mesenchymal transition (EMT), including loss of cuboidal appearance 29. As shown in Fig. 1 (A~D), TGF-β (5 ng/mL) chronic exposure or in combination with TNF-α (5, 10 ng/mL) caused an increase of sphere-forming compared with H460 cells cultured in complete medium (Fig. 1E). To further grow out the cancer stem cells from there induced cells, suspension culture system was employed 30 to select the CSCs for following experiments. As shown in Fig. F~I, the single cells from cell sphere apparently hold higher colony-forming capability and even acquired more efficiency after long term incubation in pro-inflammatory factors medium (Fig. 1J). Western blot results showed that the combined treatment of TGF-β and TNF-α could cooperatively increase the expression level of CSCs markers, CD144 and CD44 proteins (Fig. 1K, Supplementary Fig. 2). The expression level of pluripotent transcription factor Bmi1 and Oct4 also increased (Fig. 1K, Supplementary Fig. 2). In addition, TGF-β chronic exposure or in combination with TNF-α transient treatment led to upregulation of the expression of NF-κBp65 and FoxM1 (Fig. 1K). These results also showed that co-treatment of TGF-β combined with TNF-α promote the acquisition of stemness in NSCLC H460 in a dose dependent manner.

### BrMC inhibits stemness of H460 cells induced by proinflammatory cytokines

Our data here showed cytokines incubation increased the acquisition of stem cell phonotype in term of stemness. To determine whether BrMC can inhibit lung cancer stemness of H460 cells induced by proinflammatory cytokines, we used BrMC (1.0, 5.0, 10.0 μmol/L) to incubation H460 cells administered TNF-α after prolonged induction by TGF-β. As expected, BrMC effectively reduced sphere-forming (Fig. 2 A~E) and colony-forming capability (Fig. 2 F~J) induced by proinflammatory cytokines, compared with control cells. Furthermore, BrMC could downregulate the expression of CD144, CD44, Bmi1 and Oct4 (Fig. 2K, Supplementary Fig. 3). Meanwhile, BrMC notably decreased expression levels of NF-κBp65 and FoxM1 proteins, in a concentration-dependent manner (Fig. 2K, Supplementary Fig. 3). These data demonstrated that although the stemness was improved by proinflammatory cytokines treatment, BrMC can still contribute to a dose-dependent inhibition on the stemness of CSCs and downregulation of NF-κBp65 and FoxM1 expressions.

### SN50 cooperated with BrMC to inhibit stemness of H460 cells induced by proinflammatory cytokines

Activation of NF-κB involves the progression of lung cancer 17. To evaluate whether down-regulation of NF-κBp65 eliminate the increased stemness characteristics induced by proinflammatory cytokines, H460 CSCs were treated by specific inhibitor SN50 together with BrMC. Although H460 CSCs gained higher stemness characteristics (Fig. 1) by TGF-β incubation following administered TNF-α, as shown in Fig. 3, stemness characteristics were significantly reduced in presence of SN50 or BrMC. SN50 (10.0μmol/L) significantly inhibited CSCs spare (Fig. 3A~E) and colony forming capability (Fig. 3 F~J), and decreased the expression levels of CD144, CD44, Bmi1 and Oct4 (Fig. 3K, Supplementary Fig. 4). Remarkably, in combination of BrMC and SN50 enhanced the inhibition of stemness characteristics as well as down-regulation of FoxM1 expression (Fig. 3K, Supplementary Fig. 4). However, with cooperativity between downregulation of FoxM1 and BrMC affection, compared the SN50 only, the lower concentration of BrMC alone significantly inhibited stemness characteristics and reduced the expression of NF-κBp65 and FoxM1. It suggests that inhibition function of BrMC may be through downregulation of NF-κBp65 expression in H460 CSCs.

### Co-treatment of thiostrepton and BrMC cooperatively inhibited stemness of H460 cells induced by proinflammatory cytokines

Recent reports identified up-regulation of FoxM1 involved initiation of lung tumorigenesis, which raised a potential pharmacological target 31. To assess the role of FoxM1 downregulation in inhibitory effects of BrMC on stemness of H460 cells induced by proinflammatory cytokines, H460 cells administered TNF-α after prolonged induction by TGF-β were treated with thiostrepton and BrMC alone or in combination. The cooperative inhibitory effect of BrMC combined with thiostrepton on stemness of H460 cells induced by proinflammatory, including sphere-forming (Fig. 4A~E) and colony-forming capability (Fig. 4F~J) as well as expression of CD144, CD44, Bmi1 and Oct4 were shown (Fig. 4k, Supplementary Fig. 5). Interestingly, BrMC (5.0 μmol/L) and thiostrepton (10.0 μmol/L) alone or in combination significantly reduced expression of FoxM1 protein, accompanied by downregulation of NF-κBp65 expression (Fig. 4k). These results suggest that inhibitory effects of BrMC on stemness of H460 cells induced by proinflammatory cytokines may be required for downregulation of FoxM1 expression.

### Overexpression of NF-κBp65 weakens inhibitory effects of BrMC on stemness of H460 cells induced by inflammatory factors

In order to corroborate whether NF-κB expression is involved in the BrMC inhibition, CSCs after incubation of proinflammatory cytokines were used to overexpress NF-κBp65 via lentiviral vectors. With overexpression of NF-κBp65, stemness characteristics and BrMC inhibition were evaluated. As shown in Fig. 5, the overexpression of NF-κBp65 promoted the sphere (Fig. 5 A~E) and colony formation (Fig. 5 F~J), as well as increased expression of CD144, CD44, Bmi1 and Oct4 in the treated H460 CSCs (Fig. 5K, Supplementary Fig. 6). In addition, overexpression of NF-κBp65 could substantially antagonize inhibitory effects of BrMC on sphere formation (Fig. 5E), colony formation (Fig. 5J) and expression of CD144, CD44, Bmi1 and Oct4 (Fig. 5K) in H460 cells administered TNF-α after prolonged induction by TGF-β. These results indicate that inhibitory effects of BrMC on stemness of H460 cells induced by proinflammatory cytokines may be dependent on downregulation of NF-κBp65 expression.

### Overexpression of FOXM1 weakens inhibitory effects of BrMC on stemness of H460 cells induced by proinflammatory cytokines

FoxM1 is critical in the tumorigenesis, which is thought to be a potential target for inhibition the self-renewal of CSCs. In above results (Fig 1K), FoxM1 was boost by the introduction of proinflammatory cytokines in H460 cells, which may beneficial for the acquisition of stamens in CSCs. To confirm whether BrMC target to FoxM1 in the inhibition of CSCs self-renewal, lentivirus vector was employed to fulfill the overexpression of FoxM1 in H460 cells after induction by TNF-α and TGF-β. Compared to empty vector, the overexpression of FoxM1 promoted the self-renewal activity of H460 CSCs, both in the sphere formation (Fig. 6 A, C, E) and colony formation capacity (Fig. 6 F, H, J). Meanwhile, with FoxM1 overexpression, CSCs characteristics were enhanced as the stem cell markers CD144, CD44, Bmi1 and Oct4 were promoted (Fig. 6K, Supplementary Fig. 7). Specially, the NF-κB pathway was activated in the presence of raised FoxM1 abundance (Fig. 6K, Supplementary Fig. 7). As hypothesized, abnormal overexpression of FoxM1 compromised the inhibition of BrMC on stemness capacity. The efficiency of sphere formation (Fig. 6 B, D, E) and colony forming units (Fig. 6 G, I, J) was slightly recovered. In addition, overexpression of FoxM1 could reverse inhibitory function of BrMC on the expression of CD144, CD44, Bmi1 and Oct4 (Fig. 6K, Supplementary Fig. 7). These results support that down-regulation of FoxM1 expression involved the inhibitory effects of BrMC on stemness of H460 cells.

## Discussion

Studies have recently demonstrated that chronic inflammation-induced carcinogenesis and metastasis is a major challenge to cancer therapy, and elevated cytokines in chronic inflammation contribute to mortality in many malignancies, including NSCLC 32-34. Understanding the mechanisms underlying induction of the metastasis and carcinogenesis by pro-inflammatory cytokines might lead to a novel therapeutic approach 35. In this study, we first demonstrated that co-treatment of pro-inflammatory TNF-α and TGF-β cooperatively promoted lung cancer stemness of NSCLC H460 cell line via NF-κB and FoxM1. In addition, we also revealed that BrMC, a novel synthetic analogue of dietary flavonoid chrysin significantly inhibited lung cancer stemness of NSCLC H460 cell line induced by pro-inflammatory cytokines through downregulating expression of NF-κB and FoxM1 proteins. These results presented in our experimental works indicated that the bidirectional activation of NF-κB and FoxM1 not only may be a key biological marker for promotion of lung cancer stemness, but also may be a molecular target for the inhibitory effects of BrMC on lung cancer stemness of NSCLC H460 cell line induced by pro-inflammatory cytokines.

Many studies have showed that TNF-α combined with chronic exposure to TGF-β induces carcinogenesis of several tumors, including breast cancer 36 and cervical cancer 16. We have previously demonstrated that TNF-α and TGF-β associated EMT occurs via NF-κB-dependent transcriptional upregulation of Twist1. Here, we constructed the model for induction of lung cancer stemness, including elevated sphere-forming and colony forming capabilities, increased expression of CSC-associated markers (CD133 and CD44) and multipotential transcription factors (Bmi1 and Oct4) by chronic inflammation using co-treatment with TNF-α and TGF-β to NSCLC H460 cells. Our study clearly showed that H460 cells administered TNF-α after prolonged induction by TGF-β parallelly upregulated NF-κBp65 and FoxM1 protein expression. Consistently, the exposure to pro-inflammatory cytokines also leads to stemness, including sphere and colony formation, and CSC-associated protein expressions. Inhibition or overexpression of NF-κBp65 accordingly alters FoxM1 protein expression. Conversely, inhibition or overexpression of FoxM1 also accordingly alters NF-κBp65 protein expression. These results clearly demonstrate that bidirectional interaction of NF-κB with FoxM1 participates in pathogenesis of lung cancer under inflammatory microenvironment stimulated by TNF-α combined with TGF-β (Fig. 7).

It is well known that NF-κB plays a significant role in many signaling pathways including those that are involved in cancer development and progression 37. Disrupts the interplay of NF-κBp65 and FoxM1 could eradicate leukemia stem cells in chronic myelogenous leukemia. NF-κBp65 physically interacted with FoxM1, and was recruited to the FoxM1 gene promoter to increase the transcription of FoxM1 38, 39. It showed that blocking the expression of NF-ĸBp65 and FoxM1 could inhibit the invasion and migration and increase the apoptosis of cancer cells 39. Our previous data showed that 5-allyl-7-gen-difluoromethoxychrysin, a novel synthetic analogue of chrysin synergistically enhances TRAIL-mediated apoptosis in NSCLC cell line through upregulating DR5 expression 27. Recently, we have reported that BrMC effectively inhibited CSC characteristics in hepatocellular carcinoma 26. More recently, we showed that reversed M2 polarization of TAMs by inhibition of NF-κB activation 25. In this study, we found that BrMC and SN50 alone or in combination could inhibit the expression of NF-κBp65 and FoxM1, sphere and colony formation and the expression of CD133, CD44, Bmi1 and Oct4 in H460 cells induced by pro-inflammatory cytokines, whereas, overexpression of NF-ĸBp65 almost abrogated the above effects of BrMC. These results demonstrated that inhibitory effects of BrMC on stemness of H460 cells induced by proinflammatory cytokines may be dependent on downregulation of NF-κBp65 expression (Fig. 7).

An increase of expression of FoxM1 is associated with the development and progression of many cancers, including breast, liver, prostate, brain, and lung cancers, whereas the ectopic expression of the FoxM1 accelerated the development, proliferation, and tumor growth in mouse models of prostate cancer 40. Other studies showed that thiostrepton inhibited the proliferation, migration and transformation ability of breast cancer cells by down regulating FoxM1 expression 41. In this study, we observed that treatment with BrMC and thiostrepton alone or in combination could inhibit the expression of NFkB-65 and FoxM1, sphere and colony formation and the expression of CD133, CD44, Bmi1 and Oct4 in H460 cells induced by pro-inflammatory cytokines, whereas, overexpression of FoxM1 almost abolished the above effects of BrMC. These results suggest that inhibitory effects of BrMC on stemness of H460 cells induced by proinflammatory cytokines may be dependent on downregulation of FoxM1 expression.

In summary, our results suggest that inflammatory factors TNF-α and TGF-β enhance lung cancer stemness of H460 cells through NF-κB and FoxM1, and BrMC can inhibit those induced stemness through simultaneously inhibiting expression of NF-ĸB and FoxM1 (Fig. 7). BrMC is expected to become a promising candidate for the “updruggable” treatment of lung cancer.

## Supplementary Material

Supplementary figures.

## Figures and Tables

**Figure 1:** ** Co-treatment of TGF-β and TNF-α induces lung cancer stemness in H460 cells.** H460 cells were exposed to different concentrations of TNF-α (5, 10 ng/mL) for 24h following treated with TGF-β (5.0 ng/mL) for 30 d. Sphere forming rate (A~E) and colony forming rate (F~J) were evaluated. Stemness appearance was determined by lung cancer stem cell makers CD133, CD44, Bmi1 and Oct4 through western blot (K). Activation of NF-κB pathway (NF-κBp65) and human proto-oncogene FoxM1 were analyzed by western blot (K). ^*^P<0.05, *vs* untreated cells; ^#^*P*<0.05, *vs* treated with TGF-β only.

**Figure 2:** ** Effects of BrMC on stemness of H460 cells induced by pro-inflammatory cytokines.** H460 CSCs after chronic exposure to TGF-β followed by TNF-α incitation were treated with BrMC. The inhibition of BrMC was tested by cancer sphere forming (A~E) and soft ager colony forming (F~J) with single CSCs suspension. The effection on stemness capacity was evaluated by expressions of lung stem cell markers CD133, CD44, Bmi1 and Oct4 via western blot (K). The regulation on activation of NF-κB signaling and proto-oncogene FoxM1 were analyzed by western blot in CSCs under different concentrations of BrMC (1, 5, 10 μM). ^*^P<0.05, *vs* untreated cells; ^#^*P*<0.05, *vs* treated with BrMC only.

**Figure 3:** ** Effects of SN50 on inhibition of stemness of H460 cells induced by proinflammatory cytokines by BrMC.** In presence (+) or absence (-) of SN50, NF-κB signaling in H460 CSCs was regulated and inhibition of BrMC was determined. Stemness appearance of CSCs were evaluated by sphere forming assay (A~E) and colony forming assay (F~J). Expressions of CD133, CD44, Bmi1 and Oct4 as well as NF-κBp65 and FoxM1 were analyzed by western blot (K). ^*^P<0.05, *vs* untreated cells; ^#^*P*<0.05, *vs* treated cells by SN50 (10.0 μmol/L).

**Figure 4:** ** Effects of thiostrepton on inhibition of stemness of H460 cells induced by proinflammatory cytokines by BrMC.** H460 cells by administered TNF-α following chronic exposure to TGF-β were treated with thiostrepton (THI, 10.0 μmol/L) or BrMC (5.0 μmol/L) or both. Representative formed sphere (A~D) and cell colony (F~I) show the CSCs stemness capacity, and bar graph (E, J) show the rate individually. In presence (+) or absence (-) of **thiostrepton**, expressions of stem cell markers CD133, CD44, Bmi1 and Oct4 were analyzed by western blot (K). Inhibition of BrMC on CSCs was determined together with (+) or without (-) THI. Involvement of NF-κBp65 signaling and proto-oncogene FoxM1 were evaluated by WB. ^*^P<0.05, *vs* untreated cells. ^#^*P*<0.05, *vs* treated cells with THI only.

**Figure 5:** ** Effects of overexpression of NF-κBp65 on inhibition of stemness of H460 cells induced by proinflammatory cytokines by BrMC.** With chronic exposure to TGF followed by incubation of TNF-α, H460 cells were introduced NF-κBp65 by lentivirus GFP vectors. H460 CSCs expressing NF-κBp65 (+) or empty vector (-) were treated with (+) or without (-) BrMC (5.0 μmol/L). Then, those CSCs were used to perform sphere forming (A~E) in suspension culture and soft agar colony formation assay (F~J). Expressions of CD133, CD44, Bmi1 and Oct4 as well as NF-κBp65 and FoxM1 were analyzed by western blot (K). ^*^P<0.05, *vs* vector control; ^#^*P*<0.05, *vs* H460 cells with vector treated by BrMC only.

**Figure 6:** ** Effects of overexpression of FoxM1 on inhibition of stemness of H460 cells induced by proinflammatory cytokines by BrMC.** With chronic exposure to TGF followed by incubation of TNF-α, H460 cells were introduced FoxM1 by lentiviral GFP vectors. H460 CSCs expressing FoxM1 (+) or empty vector (-) were treated with (+) or without (-) BrMC (5.0 μmol/L). Sphere forming (A~E) in suspension culture and soft agar colony formation assay (F~J) with single CSCs suspension were performed to evaluate the stemness capacity. Stem cell markers CD133, CD44, Bmi1 and Oct4 were analyzed by western blot (K), as well as NF-κBp65 activity and FoxM1 expression were tested. ^*^P<0.05, *vs* vector control; ^#^*P*<0.05, *vs* H460 cells with vector treated by BrMC only.

**Figure 7:** ** Illustration of BrMC function mechanism in targeting NSCLC-CSC via NF-κB/FoxM1 signalling**. Pro-inflammatory factors TNF-α and TGF-β can promote the self-renewal capacity as well as activate NF-κB signalling in NSCLC-CSC, which also increase the expression of stem cell markers CD133, CD44, Bmi1 and Oct4. Alternatively, oncogenic transcriptional factor FoxM1 works as downstream co-activators of NF-κB signalling to increase the self-renewal capacity of NSCLC-CSC. BrMC works as inhibitor of CSC through targeting NF- κB/FoxM1 in does dependent manner.
